# Analysis on Time-Series Data from Movie Using MF-DCCA Method and Recurrent Neural Network Model Under the Internet of Things

**DOI:** 10.1155/2022/7400833

**Published:** 2022-07-08

**Authors:** Ruomu Miao, Boyuan Zhang

**Affiliations:** ^1^School of Media and Communication, Shanghai Jiao Tong University, Shanghai 200240, China; ^2^School of Music, Film, and Television, Tianjin Normal University, Tianjin 300382, China

## Abstract

The present work aims to analyze the time-series data (TSD) from movies and support constructing the movie recommendation system. Referencing the Internet of Things (IoT) technology as the framework, a time-series data analysis system for movies is built based on the recurrent neural network (RNN) and multifractal detrended mobility cross-correlation analysis (MF-DCCA) method. First, the traditional RNN model is improved by replacing the conventional convolution operation with spatial adaptive convolution. Specifically, an additional convolution layer is used to obtain the position parameters required for adaptive convolution to improve the model performance to capture the characteristics of spatial-temporal transformation. Then, the MF-DCCA method is optimized to reduce the interference of noise signals to the analysis processing of TSD from movies. Finally, the TSD analysis system is tested for performance verification. The test results indicate that the method proposed here has outstanding stability and runs smoothly. When the prediction scheme is long short-term memory (LSTM) (*L* = 20), the similarity of the LSTM (*L* = 20) network under one frame is 0.977; the similarity of the LSTM (*L* = 20) network under nine frames is 0.727. This system provides a specific idea for applying the RNN model and MF-DCCA method in analyzing TSD from movies.

## 1. Introduction

With the continuous development of Internet technologies, computers are becoming even more familiar in daily life. People can use computers to search for necessary information on the Internet. However, it is challenging to quickly find the specific information in the current network environment with a tremendous amount of data, known as information overload [1, 2]. Many researchers have researched this phenomenon and related approaches, such as the search engine, which can search information in the network resource database through the input keywords and retrieve it through a specific sorting mechanism. However, this search method also has some problems: an excess of noise in the searched results. In this case, there is a personalized recommendation system [1, 3]. The personalized recommendation system can actively provide recommendation services for users. It integrates collecting, analyzing, and predicting information and recommends projects to users according to the predicted data. Movie websites contain a large number of movie resources. However, it will take users a lot of time to manually search movies on domestic and foreign websites, or even fruitless. At present, most websites provide search engines with excellent performance to let users precisely locate target movies. This method can help users quickly find movies of interest. However, most users usually do not have a clear goal. Increasing relevant recommendation systems emerge with the increase of online videos and movies. Douban Movie is a popular online movie-sharing community in China. Users can see the movie recommendation based on user evaluation through the “movies of interest” module on the website [4].

Researchers have done much work in the automatic recommendation of movies and TV series. Qiao and Cheng [5] believed that the time-series data (TSD) were critical in the present world, which gradually accumulated with time, with high dimensions and large data scales. However, the traditional feature extraction method was inadequate for the cluster analysis of the TSD. Hence, the authors trained the import data by using the recurrent neural network (RNN) to enhance the clustering function of TSD. First, they utilized the long short-term memory (LSTM) network for the feature extraction of TSD. Then, they used the pooling technology to conduct dimensionality reduction on the output characteristics in the bottom layer of the LSTM network. Finally, they employed the imbalanced K-means algorithm to cluster the reduced-dimensionality characteristics because of the imbalance of most TSD. Meanwhile, experiments were carried out on numerous open, acquirable TSD sets. The authors found that the TSD could be efficiently treated through the combination of the dimensionality reduction via the pooling technology, the cluster analysis of imbalanced data, and feature extraction through the LSTM network. Majumdar and Laha [6] proposed a new time-series classification and clustering method based on the extension of topological data analysis technology. Zhu and Xiao [7] developed a novel precise TSD integration algorithm based on evaluation laboratory models and decision tests after discussing the relation between data. The authors validated the effectiveness and feasibility of the algorithm via numerical examples. Geng and Luo [8] reduced the influence of time intervals on fusion results by analyzing various factors in the model, combined with an ordered weight aggregation operator algorithm. Hu et al. [9] presented a straightforward and practical neural layer to normalize the input time series adaptively. The neural layer used backpropagation to train the model end-to-end, significantly improving the performance compared with other standard schemes. Unlike the traditional normalization method, this method could learn to normalize a specified task rather than utilizing a stationary normalization approach. Besides, it was suitable for any novel TSD without retraining. Le et al. [10] reported that the development of the IoT had popularized all kinds of sensors in various industrial fields and led to a massive increase in sensor data. Because of sensor data's high capacity and dimension, there is a limitation in direct deep data analysis and original DST mining of sensors. Therefore, the authors proposed a multiresolution representation and dimensionality reduction method of sensor data, using a right quantity of critical data points in a specific sensing TSD to generate the equivalent multiresolution segmented linearization portrayal. Theoretical analysis and experimental results showed that the multiresolution piecewise linear representation could reduce the dimension while keeping the critical features of TSD.

After summarizing the current situation worldwide, it is found that traditional algorithms consume a lot of time and space when performing recommendation calculations and cannot cope with the increasing number of users and items. In the past few years, deep learning has been used in image processing. Breakthroughs have been made in the field of classification and speech recognition. Artificial neural network has the characteristics of high computing power, nonlinear mapping ability, high parallelism ability, and generalization ability. As a kind of artificial neural network, convolutional neural network (CNN) has both the advantages of traditional artificial neural network and its unique advantages, so its application in the field of recommendation has important research value.

The feasibility of this study lies in that after researching some existing knowledge points, and the CNN and the RNN are combined and applied in movie rating and recommendation according to the relevant characteristics of deep learning. Finally, the structure of the two neural networks is analyzed and combined accordingly. In this paper, the user's historical rating record behavior is regarded as a sequence of information. An RNN is used to analyze the user's interest and perform corresponding modeling operations combined with the user's rating information. The information of the user and the movie is extracted by a CNN for the subsequent combination.

This paper uses the RNN model and the multifractal detrended mobility cross-correlation analysis (MF-DCCA) method to construct a TSD analysis system for movies. The research innovation lies in two aspects. On the one hand, a spatial adaptive convolution LSTM algorithm is proposed. Inspired by the spatial transformation network, this paper changes the traditional convolution operation to spatial adaptive convolution during the “input-to-state” calculation process inside the convolutional LSTM. An additional convolutional layer is utilized to obtain the position required for the adaptive convolution parameter. Then, the adaptive convolution selects the convolution position according to the spatiotemporal information and improves the model's performance to capture the spatiotemporal transformation features. On the other hand, the construction process and metrics of the MF-DCCA method are studied and used for the analysis of TSD of movies.

## 2. Analysis System of TSD from Movies

### 2.1. Optimization of LSTM Network and Construction of Internet of Things System

A neuron in the LSTM model contains a cell state and three gate mechanisms. The cell state is the basis of the LSTM model, equivalent to the model memory. The LSTM model uses the forget, update, and output gates to protect and control the cell state. The input gate controls the candidate state, the forget gate manages the information to be overlooked, and the output gate controls the output information.  Figure 1 shows the architecture of the LSTM model.

Combining LSTM with convolution operation can input image-level features into the LSTM network [11, 12]. But such a procedure does not solve the pain point of video sequence analysis in a practical sense. Only using convolution operation cannot filter the information features of the image sequence and cannot meet the performance requirements of video sequence analysis [13–15]. Therefore, researchers design an explicit processing module for the network, explicitly handling the above transformations. This paper proposes a spatial adaptive convolutional LSTM model based on the above ideas, as presented in Figure 2.

The network structure reported here is similar to the classical video prediction network structure, namely the encoder-predictor structure. The network stacks three hidden layers, i.e., the spatial adaptive convolutional LSTM layer [16, 17]. A downsampling/upsampling layer is inserted between the hidden layers. The sampling layer is essentially a convolution operation to enable the network to characterize the low-level local detail dynamics and high-level global dynamic information in a targeted manner. The network output terminal is placed at the bottom layer of the network. Therefore, high-level spatiotemporal features can guide the calibration and update of low-level local spatiotemporal features from top to bottom and use low-level state information to improve the prediction performance of details. The convolution calculation is to map the target position of the input image and the pixel information of several fixed places around it to the corresponding position of the output image. The mathematical expression of the calculation process of the 3 × 3 convolution operation is shown in.

(1) $$\begin{array}{c} y_{i,j}=\sum_{l}^{L}W_{l}\cdot x_{p_{l,i,j},q_{l,i,j}}. \end{array}$$

In equation (1), *L* represents the number of connections per point of the output relative to the input. In the traditional convolution operation with the 3 × 3 convolution kernel, *L*=9. *p*_*l*,*i*,*j*_ and *q*_*l*,*i*,*j*_ denote the location parameters of *l*th connection with the output location of (*i*, *j*).

The network structure of this paper is similar to the classical video prediction network structure, that is, the encoder-predictor structure. The network stacks three hidden layers, namely the spatially adaptive convolutional LSTM layer. Besides, a downsampling layer or an upsampling layer is inserted between the hidden layers. The sampling layer is a convolution operation, enabling the network to characterize the low-level local detail dynamics and high-level global dynamic information in a targeted manner. The network output is placed at the bottom layer of the network, so high-level spatiotemporal features can guide the calibration and update of low-level local spatiotemporal features from top to bottom and use low-level state information to improve the prediction performance of details.

In the convolutional LSTM, the objects of the convolution operation are the input of the current time step and the state variables of the previous time step. The spatial features of the input and state are extracted through the multilayer convolution operation to determine the trade-offs of state variables and input information at each spatial location. The convolution calculation is to map the target position of the input image and the pixel information of several fixed positions around it to the corresponding position of the output image. Takes the 3 × 3 convolution operation as an example. Its essence is the mapping from input to output. The pixel value of each position of the output is related to the 9 points around the corresponding position of the input. After finding the corresponding input positions of all target positions, the sum of different weights is given to different channels in the same position. Finally, the sum of the weighted results of different positions is the output.

Figure 3 demonstrates an ordinary 3 ∗ 3 convolutional neural network (CNN).

The information contained in the current time step is not necessarily the same as that in the previous time step when time and space changes are complex. Based on this, this paper does not fix the convolution kernel size. In this way, the spatial position of each convolution in the convolution operation can change with time to improve the model's ability to capture spatiotemporal correlations [18]. A spatial adaptive convolution operation is introduced, inspired by equation (1) and the spatial transformation network. First, the number of convolution connections *L* is determined. The position parameter *U*_*t*_ and *V*_*t*_ represent all the positions related to the output in the input. The input position can be found according to the corresponding position parameter. Then, each position in the output image corresponds to several places in the input image. Equations (2)∼(5) describe the new convolution equation to realize adaptive convolution.

(2) $$\begin{array}{c} f_{t}=\sigma \left(\begin{array}{c} \sum_{l=1}^{L}W_{fx}^{l}*\text{trans}\left(x_{t},{\text{U}}_{t,l},{\text{V}}_{t,l}\right)+\\ W_{fh}*h_{t-1}+b_{f} \end{array}\right), \end{array}$$

(3) $$\begin{array}{c} i_{t}=\sigma \left(\begin{array}{c} \sum_{l=1}^{L}W_{ix}^{L}*\text{trans}\left(x_{\text{t}},U_{t,l},V_{r,l}\right)+\\ W_{ih}*h_{t-1}+b_{i} \end{array}\right), \end{array}$$

(4) $$\begin{array}{c} {\tilde{C}}_{t}=\tanh\left(\begin{array}{c} \sum_{i=1}^{L}W_{cx}^{l}*\text{trans}\left(x_{t},U_{t,l},V_{t,l}\right)+\\ W_{ch}*h_{t-1}+b_{c} \end{array}\right), \end{array}$$

(5) $$\begin{array}{c} o_{t}=\sigma \left(\begin{array}{c} \sum_{i=1}^{L}W_{ox}^{l}*\text{trans}\left(x_{t},V_{t,l},U_{t,l}\right)+\\ W_{oh}*h_{t-1}+b_{o} \end{array}\right). \end{array}$$

In equations (2)∼(5), *U*_*t*,*l*_ and *V*_*t*,*l*_ represent the horizontal and vertical coordinates of the *l*th connection, respectively; *W*_*fh*_, *W*_*ih*_, *W*_*ch*_, and *W*_*oh*_ are the weights of each threshold layer obtained through training and learning. *C* stands for the number of channels of the input image. Each threshold layer has *L* weights. Therefore, the parameter quantity is *C* × *L*.

The position parameters used here need to be obtained by deep network training. Because the position parameters are discrete, the reverse derivation method cannot get the position parameters. Therefore, the bilinear difference method is introduced. Here, the coordinate of a position of the output feature is denoted as (*i*, *j*), and the convolution position input to the feature map is expressed as (*u*, *v*). The pixel value of (*u*, *v*) is determined by the bilinear difference method and then input to the convolution. Here, the pixel value calculation is expressed by “wrap”. *Y*=warp(*X*, *U*, *V*) represents the relationship among parameters. Equation (6) illustrates the mathematical relationship.

(6) $$\begin{array}{c} Y_{c,i,j}=\overset{H}{\underset{h=1}{\sum }}\overset{W}{\underset{w=1}{\sum }}X_{c,m,n}\text{max}\left(0,1-\left|i+V_{i,j}-h\right|\right)\text{max}\left(o,1-\left|j+U_{i,j}-w\right|\right). \end{array}$$

An explicit processing module is designed to learn the position parameters, as shown in.

(7) $$\begin{array}{c} U_{t},V_{t}=\gamma \left(x_{t},h_{t-1}\right). \end{array}$$

In equation (7), *x*_*t*_ represents the current time step's input and *h*_*t*−1_ refers to the hidden state of the previous time step. Besides, *γ* denotes a convolution operation between *x*_*t*_ and *h*_*t*−1_ and *U*_*t*_, *V*_*t*_ stands for the convolution output.

The traditional convolutional LSTM directly uses the image of the current time step or the output of the upper-layer convolutional RNN as the input of the present time step. In contrast, the spatial adaptive convolution LSTM reported here obtains the topological link between the output of the adaptive convolution layer and the input through the *γ* convolution operation before inputting the image. Then, it uses the topological link to spatially transform the current input to make it align with information in the hidden state for accurate memory preservation and image sequence prediction.

Aiming at the multivariate correlation characteristics of movie sequence data, this paper proposes an improved multivariate LSTM model to predict movie time series. The network structure of the model includes three layers: input layer, hidden layer, and output layer. The input layer controls the format of the input data. The hidden layer is a structure containing several LSTM units, and the error is reduced until convergence by repeated iteration and adjustment of weights. The output layer restores the results to the original data format. The input layer converts the preprocessed time-series data into data that can be used for supervised learning. *T* time steps are selected as intervals, the data of *T* time steps before each moment are taken as the input of this moment, and the corresponding sample value of this moment is taken as the target output. The data are divided into input sets and corresponding output sets. This paper integrates multitype sensor data into 3-dimensional data: [sample value, time step, feature] to make the input data contain multivariate. The input is then entered into the hidden layer with a time step as the unique index.

This paper examines the cross-correlation between Google search volume for financial keywords and movie box office. Multifractal features including the coronavirus disease 2019 (COVID-19) period and before the COVID-19 outbreak are discussed. The dynamic evolution of cross-correlation and the impact of COVID-19 on the cross-correlation between the film industry and financial market volatility are observed through the sliding window method. Using the MF-DCCA method, this paper reveals the cross-correlation between two emotion proxies: Google Trends' fear index and Twitter's daily happiness index.

Earlier researchers defined the Internet of Things (IoT) as a network connecting everything to the Internet to solve the connection between people and things and items and things. The study summarizes the IoT as an intelligent network consisting of perception, network, and application layers to connect people and things or things and things. The essence of IoT is to complete the interaction and connection between people and things or items and things. People or things can control things through the network, and the corresponding things can receive control signals and generate related actions. At present, the functions of the IoT are constantly expanding and updating, evolving from simple object positioning, tracking, and evolution to applying various sensors and intelligent information processing technologies. Like traditional IoT, the polymorphic IoT also has three layers: perception layer, network layer, and application layer. However, it can collect more comprehensive information than traditional IoT. Besides, its network layers also become more complicated when processing data. In polymorphic IoT, the primary vital technologies include radio frequency identification (RFID) and wireless network sensor technology. This paper believes IoT is an extension based on the Internet with the same foundation. The user end of the IoT can expand to anyone and objects [19, 20].  Figure 4 displays the service-oriented architecture (SoA) structure of IoT.

SoA in IoT is necessary for service users and providers. SoA guarantees the interoperability between heterogeneous devices in several ways.  Figure 4 provides a common SoA consisting of four layers with different functions. (1) Data perception layer: the perception layer integrates with valid hardware targets to perceive the state of things. The perception layer contains terminals collecting data from IoT, including RFID tags, intelligent phone terminals, wireless sensors, and Bluetooth. (2) Network layer: it is the infrastructure supported by wireless or wired links. The network layer in IoT links everything and enables them to perceive their ambience. Things can share data with interconnected objects through the network layer, essential for intelligent event processing and management in IoT. In addition, the network layer can gather data from current IT infrastructure and then transfer the data to high-level decision-making units, complex services. (3) Service Layer: the service layer is the services required to manage and create applications or users. The service layer needs the support of middleware technology, a crucial initiator of IoT applications and services. Middleware technology offers a cost-efficient system that can reuse hardware and software platforms. (4) Interface layer: the interface layer is composed of the interactive modes with the user or application. In IoT, there are many devices provided by different vendors. Thus, the interface layer does not always adhere to the same standard. Through the previous introduction to the basic architecture of the IoT, the TSD of IoT analyzed here principally comes from the data perception layer. This paper concludes the following characteristics of the TSD of IoT from analyzing the devices with multitudes of data perception layers. (1) Massive: in such a vast IoT architecture, the terminals generate and transmit data all the time. (2) High frequency: these IoT sensing terminals have a very high sensing frequency to monitor and sense the surrounding environment at all times. (3) Heterogeneity: since data streams come from many spatially distributed data sources, IoT data are of different kinds. Also, since mobile devices in the perception layer support multiple sensors, they have different data types. (4) Time dependence: it has a strong temporal correlation. IoT sensor data collected by devices placed in specific locations are time stamped.

### 2.2. Multifractal Analysis Method of Time Series

With the deepening of research on nonlinear theory, researchers have put forward many methods for multifractal analysis of time series. In the 1990s, Shen et al. proposed the trended fluctuation analysis method. Gil et al. put forward the multifractal detrended fluctuation analysis (MF-DFA) method based on Shen et al., which could easily calculate the main parameters of time series [21, 22]. The conventional Euclidean geometry cannot describe complicated atypical objects in nature. Correspondingly, the concept of fractal was born in the 1960s, indicating the erose objects. The contour lines of the fractal are represented by anomalous fractal curves. There is only a descriptive definition of a fractal without a mathematical description [23, 24]. The generally represented fractal has five features. (1) The fractal is a small-scale complicated and delicate configuration. (2) Conventional geometric expression cannot describe it in a direct manner. (3) It has statistical self-similarity and approximate self-similarity. (4) The fractal dimension is more than the topological dimension in some cases. (5) Recursive methods can produce plain fractal pictures. The categorical attributes can be discussed from two aspects based on the classification characteristics. On the one hand, it is essential to judge whether there is a “scale space.” The same natural phenomenon has several scale-free intervals under specific conditions according to the relevant research data. The fractal characteristics may differ in different scale intervals. On the other hand, fractal inlay in nature is the opposite of that in mathematics. The following fractals in the present work belong to the mathematical sense. Generally speaking, the rationale and practical use of fractal are studied in a theoretical perfect space, named the fractal space [25, 26]. The *q* fluctuation function *F*_*q*_(*s*) in the multifractal detrended fluctuation analysis algorithm can be written as.

(8) $$\begin{array}{c} F_{q}\left(s\right)={\left\{\frac{1}{2N_{s}}\overset{2N_{s}}{\underset{v=1}{\sum }}{\left[F^{2}\left(s,v\right)\right]}^{\frac{q}{2}}\right\}}^{1/q}. \end{array}$$

In equation (8), *q* is any real number that is not zero; *F*_*q*_(*s*) increases with the growth of *s* in a power-law relationship. For each *s*, there is a corresponding function value *F*_*q*_(*s*).

The detrended cross-correlation analysis method analyzes the power-law long-term interrelation among different nonstationary time series. For two time series, *F*2(*s*) and the sum scale *s* obey the power-law relationship *F*2(*s*) ~ *sλ* in double logarithmic coordinates. *λ* means the long-term inter-relation scale coefficient. *λ* > 0.5 signifies the positive long-term inter-relation between the two series and vice versa [27, 28]. The DCCA method can be extended to study the long-term inter-relation between two unsteady signals. It is assumed that there are two time series denoted as {*x*(*t*)} and {*y*(*t*)}, where *i*=1, −2,3 …, *M*. The mean values of the two time series are 0, and the time series is composed of *M*_*s*_=(*M*/*s*) blocks with a nonoverlapping size of *s*. The *𝒱*_*th*_ block [*l*_*v*_+1, *l*_*v*_+*s*] can be written as equations (9) and (10).

(9) $$\begin{array}{c} X_{v}\left(k\right)=\overset{k}{\underset{j=1}{\sum }}x\left(l_{v}+j\right), \end{array}$$

(10) $$\begin{array}{c} Y_{v}\left(k\right)=\overset{k}{\underset{j=1}{\sum }}y\left(l_{v}+j\right),\;k=1,\ldots ,s. \end{array}$$

The local tendencies of {*Y*_*v*_(*k*)} and {*X*_*v*_(*k*)} are expressed by

$\left\{{\tilde{Y}}_{v}\left(k\right)\right\}$ and $\left\{{\tilde{X}}_{v}\left(k\right)\right\}$. Equation (11) illustrates the trend covariance of each block.

(11) $$\begin{array}{c} F_{v}\left(s\right)=\frac{1}{s}\overset{s}{\underset{k=1}{\sum }}\left[X_{v}\left(k\right)-X_{v}\left(k\right)\right]\left[Y_{v}\left(k\right)-{\tilde{Y}}_{v}\left(k\right)\right]. \end{array}$$

When *q*=0, the *q*_*th*_ detrended covariance can be written as.

(12) $$\begin{array}{c} F_{xy}\left(q,s\right)={\left(\frac{1}{m}\overset{m}{\underset{v=1}{\sum }}F_{v}{\left(s\right)}^{q/2}\right)}^{1/q}. \end{array}$$

When *q*=0, the *q*_*th*_ detrended covariance can be expressed as.

(13) $$\begin{array}{c} F_{xy}\left(0,s\right)=\exp\left(\frac{1}{2m}\overset{m}{\underset{v=1}{\sum }}\ln\;F_{v}\left(s\right)\right). \end{array}$$

Equation (19) can be transformed into.

(14) $$\begin{array}{c} F_{xy}\left(q,s\right)∼s^{h_{xy}\left(q\right)}. \end{array}$$

To sum up, the calculation process of the DCCA method can be divided into five steps. First, two time series are defined as {*x*_*t*_} and {*y*_*t*_}, (*t*=1,2 …, *N*) with time length of *N*.

(1) Two new time series are established on the basis of {*x*_*t*_} and {*y*_*t*_}, (*t*=1,2 …, *N*), as shown in.
  (15) $$\begin{array}{c} X\left(t\right)=\sum_{i=1}^{t}\left[x_{i}-\langle x\rangle \right],\\ Y\left(t\right)=\sum_{i=1}^{t}\left[y_{i}-\langle y\rangle \right]. \end{array}$$
In equation (15), 〈*x*〉 and 〈*y*〉 represent the average value of {*x*_*t*_} and {*y*_*t*_}, (*t*=1,2 …, *N*).
(2) Y(*t*) and X(*t*) are separated into subtime series without crossing with the number of *N*_*s*_=[*N*/*S*].
(3) The local trends *X*_*v*_(*i*) and *Y*_*v*_(*i*) of the time series are evaluated by the least square method. Then, the downward trend covariance *F*^2^ is obtained, as shown in.
  (16) $$\begin{array}{c} F^{2}\left(s,v\right)=\frac{1}{s}\overset{s}{\underset{i=1}{\sum }}\left|Yvs-Ys+Yi-Y_{v}\left(i\right)\right|\cdot \left|Xvs-Xs+Xi-X_{v}\left(i\right)\right|. \end{array}$$
For each subtime series *v*(*v*=1,2 …, *N*_*s*_), there is the relationship shown in.
  (17) $$\begin{array}{c} F^{2}\left(s,v\right)=\frac{1}{s}\overset{3}{\underset{i=1}{\sum }}\left|YN-Yv\text{S}+YN_{s}s+Yi-Y_{v}\left(i\right)\right|\cdot \left|XN-Xvs+XN_{s}s+Xi-X_{v}\left(i\right)\right|. \end{array}$$
(4) The downward trend covariance function of the whole time series is obtained by taking the average value of the downward trend covariance of the subtime series with the number of 2*N*_*s*_, as presented in.
  (18) $$\begin{array}{c} {\text{FF}}_{DCCADCCA}^{2}2^{2}\left(s\right)=\frac{1}{2N_{s}}\overset{2N_{s}}{\underset{v=1}{\sum }}F^{2}\left(s,v\right). \end{array}$$
(5) There is a power-law correlation between the downtrend covariance function *F*_*DC*  *CA*_(*s*) and the time scale *s*, as shown in.
  (19) $$\begin{array}{c} {\text{F}}_{DCCA}\left(s\right)\propto s^{h}. \end{array}$$
In equation (19), *h* means the thurst index.
The MF-DFA method's calculation process is like the detrended fluctuation analysis approach, except for Step 4. Equation (20) demonstrates Step 4 of MF-DFA.
Equation (20) manifests the decreasing trend variance function with *q* order of time series when *q*=0.
  (20) $$\begin{array}{c} F\left(q,s\right)={\left\{\frac{1}{2N_{s}}\overset{2N_{s}}{\underset{v=1}{\sum }}{\left[F^{2}\left(s,v\right)\right]}^{q/2}\right\}}^{1/q}. \end{array}$$
When *q*=0, there is a relationship as shown in.
  (21) $$\begin{array}{c} F\left(q,s\right)=exp\left\{\frac{1}{4N_{s}}\overset{2N_{s}}{\underset{v=1}{\sum }}\ln\left[F^{2}\left(s,v\right)\right]\right\}. \end{array}$$

## 3. Experimental Environment and Experimental Data set Configuration

Table 1 lists the hardware and software environment in this experiment.

Mixed National Institute of Standards and Technology (MNIST) is a picture data set of handwritten numbers. The data set was organized by the National Institute of Standards and Technology in the United States, counting a total of 250 pictures of handwritten numbers by different people. It is also a basic data set in the field of computer vision. Many projects related to computer vision conduct basic experiments on this data set.

The experimental data set used here is the MNIST data set. There are 60,000 pictures in the MNIST data set. This paper uses 80% of the pictures as the training set and the rest as the test set. In this paper, the data in the training set are composed of 40,000 image sequences with a length of 25 frames, and the pictures in the test set are composed of 20,000 image sequences with a length of 25 frames. This paper randomly selects 3 numbers from 0 to 9 and then selects the corresponding digital pictures from the MNIST data set. The material rotation angle and zoom factor are set to generate 20 frames of video. This paper also uses the public movie data set MovieLens for training. The data set contains three parts: user data, movie data, and user rating data. The user data include user identification (ID), user gender, user occupation, user age, and the code of the user's region. Since the code of the location region can only represent the region to which the user belongs, the scope is very wide and cannot be representative, so this attribute is eliminated. Movie data contain movie ID, movie name, and movie genre. It should be noted that the movie name field is a combination of the movie name and the release time. There are a total of 18 movie genres. A movie may belong to more than one movie genre. User rating data are composed of user ID, movie ID, rating, and timestamp.

In the model's training process, the Adam algorithm is used to optimize this model. The data set constructed via the MNIST database is used to train the network. The network is set to iterate 1,500 times. Control variables are used to verify the effectiveness of the optimized algorithm after all iterations. Batch size will affect two aspects of the network: the optimization performance and the convergence speed of the model and the memory size of the GPU. When the value of batch size is enormous, the convergence speed of the model becomes fast, but the increase of accuracy is reduced to some extent. After many experiments, this paper set the batch size to 8. This experiment tests the three layers adaptive convolution LSTM. The number of convolution kernels in each threshold layer from bottom to top is 64, 192, and 192, respectively.

## 4. Algorithm Test and Simulation

### 4.1. System Test

Table 2 summarizes the test results of the common user function and the system administrator function.

As can be seen from Table 2, when the system performs the function test of ordinary users, all the subfunction tests of the system pass. When the system performs the function test of the system administrator, all the subfunction tests of the system pass. To sum up, the system has good stability, and the functions of this part meet the analysis requirements.

Figure 5 presents the pressure test results of the system, in which the abscissa refers to the number of users, and the ordinate refers to the worst-case response time.

The difference between the two tests in Figure 5 is that the environment for the first test is relatively simple, and the environment for the second test is complex. The system stress test results indicate that the system's response time rises with increased user concurrency. When the user concurrency is 10, the worst-case response time of the request is 0.634 s, the mean response time of the proposal is 0.342 s, and the request success rate is 100%. When the user concurrency is 500, the worst-case response time of the request is 1.342 s, the mean response time of the proposal is 0.875 s, and the request success rate is 100%. When the user concurrency is 5000, the worst-case response time of the request is 5.965 s, the mean response time of the request is 2.645 s, and the request success rate is 100%. When the user concurrency is 8000, the worst-case response time of the request is 6.233 s, the mean response time of the request is 3.174 s, and the request success rate is 100%. On the whole, although the system response time rises slightly with the increasing in users, the system can respond within the range that users can tolerate, so the performance of the system is good.

### 4.2. Frame-by-Frame Structure Similarity Evaluation of MNIST Video Prediction

Figure 6 reveals the frame-by-frame structure similarity evaluation results of MNIST video prediction, in which the abscissa is the frame time, and the ordinate is the similarity.

According to Figure 6, when the prediction scheme is PredNet, the similarity of PredNet is 0.978 under one frame; the similarity of the PredNet network is 0.206 under nine frames. In contrast, when the prediction scheme is LSTM, the similarity of the LSTM network is 0.935 under one frame; the similarity of the LSTM network is 0.551 under nine frames. When the prediction scheme is LSTM (*l* = 10), the similarity of the LSTM (10) network is 0.966 under one frame; the similarity of the LSTM (10) network is 0.707 under nine frames. When the prediction scheme is LSTM (*l* = 20), the similarity of the LSTM (*l* = 20) network is 0.977 under one frame; the similarity of the LSTM (*l* = 20) network is 0.727 under nine frames. To sum up, because PredNet lacks the Ground Truth structure to calculate the error, the similarity drops rapidly from the second frame of prediction. On the contrary, the performance of the model reported here is excellent.

Figure 7 signifies the experimental results of MNIST. The first column displays the experimental results of predicting the 2nd frame in the video sequence. The second column presents the experimental results of predicting the 10th frame in the video sequence. The third column bespeaks the prediction results of predicting the 15th frame in the video sequence.

Figure 7 suggests that when the traditional LSTM network processes an image with a complex shape, the definition of the image decreases. Still, the adaptive LSTM networks with ten links and 20 links can reasonably predict the difficult changes of the image. Compared with the adaptive LSTM network with 20 links, the adaptive LSTM network with ten links can better maintain the definition of the image, and it can better predict the clarity of the image.

## 5. Conclusions

Based on the IoT technology, an analysis system of TSD from a movie is constructed based on RNN and the MF-DCCA method. In optimizing RNN, a spatial transformation layer is added to its network structure to explicitly learn spatial-temporal changes' characteristic. The performance of the model based on cyclic neural network and MF-DCCA method is evaluated by the prediction results of handwritten video clips. Experiments show that in some cases, designing a single module to explicitly learn some features can endow the network with brilliant generalization capability. In the experiment, when the user concurrency is 5,000, the worst-case response time is 5.965, the mean response time is 2.645, and the request success rate is 100%. Adopting LSTM (*L* = 20) as the prediction scheme, the similarity of the LSTM (*L* = 20) network is 0.977 under one frame, and it is 0.727 under nine frames. Although the optimized LSTM network has considerable performance improvement compared with the traditional convolution LSTM and a strong ability to capture complex spatial-temporal variation characteristics and is more competent for the task of pixel-level video prediction. Still, it has some shortcomings. The data set used in this experiment has a small volume and simple construction. In addition, the network structure also has some room for refinement. The future work will introduce the attention mechanism into the network to enhance the prediction accuracy.

## Figures and Tables

**Figure 1:** Structure of LSTM model. In Figure 1, *T* means take, *A* represents add, *F* denotes forget the door, *U* means update the door, and *O* indicates output the door.

**Figure 2:** Spatially adaptive convolution LSTM network model.

**Figure 3:** An ordinary 3 ∗ 3 CNN. In Figure 3, *I* represents the number of channels.

**Figure 4:** Structure of SoA ((a) overall architecture; (b) detail architecture).

**Figure 5:** System pressure test ((a) 1st test; (b) 2nd test).

**Figure 6:** Frame by frame structural similarity evaluation results of video prediction on MNIST database ((a) the learning rate is 0.05; (b) the learning rate is 0.005).

**Figure 7:** MNIST experimental results ((a) test on the number “3”; (b) test on the number “5”).

**Table 1:** Settings of the hardware and software environment.

Hardware		Software	
CPU	Inter(R) core(TM)I5–7200U CPU@2.5 GHz	Database	MySQL

Operating system	Window10 64 bit ubuntu	Development framework	TensorFlow

**Table 2:** Test results of the common user function and the system administrator function.

		Number of tests	Number of failures	Success times	Pass or not
General user function test	Information update	100	0	100	Adopt
	Watch movies	100	1	99	Adopt
	Movie evaluation	100	0	100	Adopt
	Delete comments	100	0	100	Adopt
	Verification code acquisition	100	1	99	Adopt

System administrator function test	Information management	100	0	100	Adopt
	Search for movies	100	1	99	Adopt
	Update movie	100	0	100	Adopt
	Add movie	100	0	100	Adopt
	Delete movie	100	1	99	Adopt
	Log movie	100	0	100	Adopt

^*∗*^the experiments in Table 2 are similar to the experimental settings in reference [29].

## Data Availability

The data used to support the findings of this study are included within the article.
